# Study on Vertical Joint Performance of Single-Faced Superposed Shear Wall Based on Finite Element Analysis and Calculation

**DOI:** 10.1155/2022/2418874

**Published:** 2022-07-18

**Authors:** Gao-Ni Fang, Rong-Cheng Hou, Wei Ma, Kai Xu

**Affiliations:** School of Civil Engineering, Anhui Jianzhu University, Hefei 230601, China

## Abstract

In this paper, a new type of single-faced superposed shear wall system is proposed based on the single-faced superposed shear wall structure. The nonlinear finite element analysis of a new splicing form of single-faced superposed shear wall components is carried out by using the method of combining experimental research and ABAQUS finite element software analysis. The impact of noncolumn on the connection performance of vertical seam is studied. The analysis shows no significant difference in the effect of eliminating concealed column on the hysteretic performance and bearing capacity of the single-faced superposed shear wall with the joint. The single-faced composite shear wall with two different splicing forms presents bending-shear failure. The single-faced composite shear wall model without concealed column design can also maintain good overall performance and seismic behavior.

## 1. Introduction

The composite plate shear wall structure is an integral shear wall structure formed by taking the prefabricated wall as the template and pouring concrete in the inner cavity. Compared with the ordinary reinforced concrete wall, the composite shear wall has the advantages of light weight, short construction period, and good benefits. Because of its good overall performance and shear capacity, it has become the focus of attention of Chinese and foreign scholars [1–4].

Considering the structural difference between domestic and foreign superposed shear walls, many researchers did many tests to survey their axial and eccentric compression performances, out-of-plane flexural performances, and shear connector performances [5–8], whereas rare studies involved their seismic behaviors.

Most parts of China have seismic fortification requirements, so it is very important to consider the seismic performance of composite shear walls. Zhang et al. [9] conducted low-frequency cyclic horizontal loading tests at 6 horizontal connection nodes of double-faced superposed shear walls and 2 cast-in-situ nodes. Their test results indicate that the vertical joint of double-faced superposed shear walls had seismic behavior similar to the cast-in-situ nodes. However, the seismic behavior of the horizontal joint was not mentioned. Zhao et al. [10] carried out the same tests on 3 pieces of double-faced superposed shear walls, with results as shown below. When the depth-width ratio was 2.0 and the axial compression ratios were 0.2 and 0.1, increasing the area of the longitudinal joint bar effectively controlled the deformation in the bottom joint area and the damage concentration on the wall, resulting in a full and strong energy dissipation loop. Based on this result, they pointed out that joint bars can be added to improve the joint performance of superposed shear walls. H. Li and B. Li [11] surveyed the forces on 9 pieces of reinforced concrete shear walls under cyclic loading, proposed a multispring macro finite element model of the reinforced concrete shear wall, obtained a more suitable constitutive model reflecting the relationship between load and displacement, and provided the applicable calculation formula.

Because of the structural stability, industrial production, and many other advantages, the single-sided laminated plate shear wall with an insulation layer has attracted the attention of many scholars. Einea et al. [12] found that the overall performance is equivalent to that of the integrally cast concrete wall by studying the solid concrete or metal truss reinforcement as the shear transfer mode. Benayoune et al. [13] found that when the specimen is damaged, only the top or bottom concrete is damaged, and the integrity is good. Ma et al. [14] tested the seismic behavior of such shear wall, obtaining the following results: the failures of single-faced superposed slab shear wall and holistically cast-in-situ shear wall were both bending-shear failures; in the failure stage, the former structure had a little poor ductility but performed well in energy dissipation. Their research did not investigate the performance of single-faced superposed slab shear walls that were horizontally joined. However, the horizontal joint of superposed walls is inevitable in practical engineering since the dimensions of the prefabricated walls are restricted by the modes of transportation and hoisting. Ma et al. [15] got two wall slabs jointed horizontally by using embedded columns and tested the structure's seismic behavior. The results reveal that the failure form of single-faced superposed slab shear walls jointed by embedded columns and that of a holistic single-faced superposed slab shear wall were both bending-shear failures. The two structures had similar seismic characteristics properties such as hysteretic performance, ductility, and energy dissipation capacity. However, the embedded columns reduce the assembly efficiency, so there is still room for optimization of the connection form of vertical connection joints of composite plate shear walls.

This paper proposes a new type of single-faced superposed slab shear walls with joints but without embedded columns, and based on applicable tests, a finite element model is established and analyzed numerically [16–19]. Furthermore, the seismic behavior of the joint is analyzed based on a comparison of the joints' bearing capacity and failure form under low-frequency cyclic loading.

## 2. Test Overview

### 2.1. Test Design

In this test, the authors designed a test piece PJ-1 and a test piece ZT-1, with design details as presented in Figure 1. The former was two pieces of single-faced superposed slab shear walls jointed horizontally, with columns embedded at the joints, while the latter was a holistic piece of single-faced superposed slab shear wall without joint. The two test pieces had the same physical dimensions and were both composed of three parts: the base, single-faced superposed slabs, and the top beam. The mechanical properties of the main materials of the reinforcement and concrete are listed in Tables 1 and 2.

### 2.2. Loading Scheme

This test was carried out in the Anhui Provincial Key Laboratory of Building Structure and Underground Engineering. The designed axial compression ratio was 0.1. An oil Jack was applied to the top parts of the test pieces with a constant vertical load of 600 kN. The top beams were under low-frequency horizontal cyclic loading from a 100 T electro-hydraulic servo actuator to do pseudo-static tests. The loading device is illustrated in Figure 2.

The loading protocols in Figure 3 were formulated as per the *Standard for Test Method of Concrete Structures*, and the loading was under mixed control of load and displacement. In the first stage, the load is loaded through load control. The horizontal force is loaded from 50 kN and added to the specimen yield with 25 kN as the level difference. The load cycle of each level is once. After the specimen yield, the load is controlled by displacement. The multiple of the horizontal displacement value measured by the external displacement meter on the top of the shear wall and the built-in displacement meter in the system is selected for loading step by step, and each level of displacement is cycled three times. When the test piece is loaded to its own destruction or the load value of the test piece drops to 85% of the maximum load value, the test is completed.

### 2.3. Test Results

The failures on the test pieces are depicted in Figure 4. The wall edge showed horizontal cracks, as seen on test pieces PJ-1 and ZT-1. As the load increased, some horizontal cracks gradually extended and formed inclined bending-shear cracks. The inclined cracks ran at 45° roughly and finally formed X-shaped cracks. As observed from the development process and distribution of the cracks, the test pieces bent first and then sheared, forming bending-shear failures. The upper parts of the walls were almost intact, and the concrete at two ends of the base became weak and peeled off. During the entire loading on test piece PJ-1, there is no slip in the joint of the concealed column all the time, and the crack development is relatively sufficient, indicating that the joint structure of concealed column is reasonable, which can effectively splice two single-sided superimposed shear walls to form an overall common stress.

As for the hysteretic curves of the test pieces in Figure 5, their envelope areas were both in a straight line in the initial stage of loading and nearly coincided before cracking, complying with the force characteristics in the elastic stage. After yielding, the envelope areas enlarged gradually, and the test pieces' energy dissipation capacity increased somewhat. Over a comparison, it can be seen that the hysteretic curves of test pieces PJ-1 and ZT-1 almost coincided. This result implies that a vertical joint had a small impact on the hysteretic performance of a single-faced superposed slab shear wall. At the same time, the embedded columns enabled the jointed single-faced superposed slab shear walls to form a whole part subjecting to a holistic force.

## 3. Calculation for the Finite Element Analytical Model

### 3.1. About the Model

According to the test results, the authors raised a test piece PJ-2 with the same design as PJ-1 but without embedded columns. Based on this new design, two shear-wall finite element models were established by using the Abaqus FEA.

### 3.2. Parameters of the Model

Given the loading protocols and the cyclic loading on concrete, the constitutive model of the concrete material adopted the concrete damaged plasticity model contained in the Abaqus FEA. Tensile and compression damage factors were used to depict the degradation in the initial elasticity of concrete and the damage accumulation [20]. The material properties of the model were input as per the *Code for Design of Concrete Structures* (GB50010–2010). In the finite element model, the concrete adopted the C3D8R solid element, the dilation angle was 30°, the flow eccentricity was 0.1, (*f*_*b*_0__/*f*_*c*_0__)= 1.16 (*f*_*b*_0__ is the biaxial compressive strength of concrete, and *f*_*c*_0__ is the uniaxial compressive strength), the Poisson's ratio was 0.2, the elastic modulus was 3 × 10^4^ MPa, the ratio of second stress invariants on the tensile and compression meridians was 0.667, and the viscosity coefficient was 0.005. The reinforcement adopted the T3D2 truss element. The experimental values of materials expressed the constitutive relation of concrete in the test, where the yield strength *f*_*y*_ of steel was 530 MPa, the Poisson's ratio was 0.3, and the elastic modulus was 2 × 10^5^ MPa. As the forces on the top beam and the base were not considered in the test, the two parts were designed with infinite rigid beams under ideal conditions.

The coupling points were arranged in the center of the bottom beam and fixed on the “load” module. The reinforcement got in contact with and constrained by the concrete by an embedding range constraint order. The superposed interface between the prefabricated member and cast-in-situ concrete was in binding contact. As this model was mainly used to investigate the seismic behavior of the shear wall, the interfaces between the shear wall and the loading beam and between that and the base were also arranged in binding contact. An FRP connection was set between the outer leaf board and the load-carrying wall of the test piece and bore no force all the way. For this reason, frictional contacts (friction coefficient: 0.6 [9]) were designed between the thermal insulation board and the outer leaf board concrete and between that and the post-cast intracavity concrete. The normal force transmission between the new and old superposed concrete faces was by hard contact so that the applied force vertical to the interface was fully transmitted in the cross section.

The model was designed with three analytical steps: initial step, step 1, and step 2. In the initial step, relevant boundary conditions were set. In step 1, 600 kN axial pressure was loaded at the coupling point in the center of the top beam. In step 2, the loading time was set as per the loading protocols for the test, and the load-displacement mixed control loading was simulated and converted into displacement loading based on the model's amplitude function. After conversion, the loading protocols are illustrated in Figure 6.

## 4. The Simulated Results and Analysis

### 4.1. Damage

Figures 7 and 8 display the concrete analysis results of the finite element model. As can be observed from the concrete damage cloud chart, the concrete damage at the joint of the shear wall model without embedded columns was greater than that with embedded columns. However, the two designs show almost identical holistic failure forms. According to the cloud chart of reinforcement stress, in both of the two models, the reinforcement stress on the two sides was the highest, gradually decreased toward the joint, and had no interruption and sudden change at the joint. This result demonstrates that the reinforcement meshes of both two models (with and without embedded columns) can form holistic force-bearing bodies. The reinforcement stress at the joint of test piece PJ-1 was 440.531 MPa, while that at the joint of test piece PJ-2 was 463.285 MPa, with a difference of 5.2% from the former. This result reveals that the design with or without embedded columns had no great impact on the model, and the model without embedded columns still had a good holistic performance.

### 4.2. Hysteretic Performance

As presented in the hysteretic curves and skeleton curves (Figures 9 and 10) of the two test pieces obtained by simulated calculation, the area enveloped by the hysteretic loop of PJ-2 was slightly larger than that of PJ-1. The reason was that, without embedded columns, the concrete at the vertical joint showed failures under the action of the horizontal load, so the test piece was divided into two small shear walls bearing forces continuously. At this point, the test piece has lost overall rigidity, gained ductility, and gained energy dissipation capacity. Moreover, the PJ-2's ultimate bearing capacity became a little higher than the PJ-1's. These results verify that the design without embedded columns is feasible.

As also presented in the following figures, the skeleton curves of PJ-1 and PJ-2 had similar trends. The simulated curves of the two in the elastic stage almost coincided because no significant changes occurred in the mechanical properties of the two shear walls in this stage. After entering the elastic-plastic stage with continuous loading, the reinforcement inside the test piece yielded gradually, and both the two models experienced obvious rigidity degradation. However, PJ-2's rigidity degraded more significantly than PJ-1's due to the concrete failures at the joint of PJ-2. The skeleton curves tended to be gentle in the plastic stage, which suggests that both structures had good ductility (without a large difference) after subjecting to the ultimate load.

## 5. Conclusion

In this study, the test and ABAQUS FEA were used to make finite element analysis on new single-faced superposed slab shear walls, obtaining the following conclusions:

First, the design with or without embedded columns has no significant impact on the bearing capacity and hysteretic performance of single-faced superposed slab shear walls horizontally jointed. Using the two designs, the single-faced superposed slab shear walls showed bending-shear failures. This result indicates that the horizontally jointed single-faced superposed slab shear walls with loading beam can still have good holistic performance and seismic behavior in practical engineering, even without embedded columns.

Second, the design without embedded columns helps simplify the construction process and improve assembly efficiency while ensuring the structure's bearing capacity.

Third, the optimized design was just simulated in this study and still requires further experiments in the future to verify its rationality and consistency.

## Figures and Tables

**Figure 1:** Physical dimensions and reinforcements of the test pieces. (a) PJ-1. (b) ZT-1.

**Figure 2:** Loading device for the test pieces.

**Figure 3:** The loading protocols. (a) PJ-1. (b) ZT-1.

**Figure 4:** Failures on the test pieces. (a) PJ-1. (b) ZT-1.

**Figure 5:** Hysteretic curves of the test pieces. (a) PJ-1. (b) ZJ-1.

**Figure 6:** The loading protocols.

**Figure 7:** The cloud chart of concrete damage. (a) The design with embedded columns (PJ-1). (b) The design without embedded columns (PJ-2).

**Figure 8:** The cloud chart of reinforcement stress. (a) The design with embedded columns (PJ-1). (b) The design without embedded columns (PJ-2).

**Figure 9:** Comparison of the hysteretic curves.

**Figure 10:** Comparison of the skeleton curves.

**Table 1:** Mechanical properties of reinforcement materials.

Pieces number	Reinforcement type	Diameter (mm)	Yield strength *f*_*y*_ (MPa)	Tensile strength *f*_*u*_ (MPa)	Elongation *A* (%)
PJ-1	HRB400	10	492.2	525.1	11.9
	HRB400	12	544.2	668.2	12.5

ZT-1	HRB400	10	535.6	668.5	20.01
	HRB400	12	487.3	641.2	19.03

**Table 2:** Mechanical properties of concrete materials.

Pieces number	Part	Cubic strength *f*_*cu*_ (MPa)
PJ-1	Prefabricated part	33.5
	Cast-in-place part	33.3
ZT-1	Prefabricated part	33.5
	Cast-in-place part	31.8

## Data Availability

No data were used to support this study.
